# An Approach for Thoracic Syndrome Classification with Convolutional Neural Networks

**DOI:** 10.1155/2021/3900254

**Published:** 2021-09-21

**Authors:** Sapna Juneja, Abhinav Juneja, Gaurav Dhiman, Sanchit Behl, Sandeep Kautish

**Affiliations:** ^1^IMS Engineering College, Ghaziabad, India; ^2^KIET Group of Institutions, Delhi NCR, Ghaziabad, India; ^3^Govt. Bikram College of Commerce, Patiala, India; ^4^BMIET, Sonepat, India; ^5^LBEF Campus, Kathmandu, Nepal

## Abstract

There have been remarkable changes in our lives and the way we perceive the world with advances in computing technology. Healthcare sector is evolving with the intervention of the latest computer-driven technology and has made a remarkable change in the diagnosis and treatment of various diseases. Due to many governing factors including air pollution, there is a rapid rise in chest-related diseases and the number of such patients is rising at an alarming rate. In this research work, we have employed machine learning approach for the detecting various chest-related problems using convolutional neural networks (CNN) on an open dataset of chest X-rays. The method has an edge over the traditional approaches for image segmentation including thresholding, *k*-means clustering, and edge detection. The CNN cannot scan and process the whole image at an instant; it needs to recursively scan small pixel spots until it has scanned the whole image. Spatial transformation layers and VGG19 have been used for the purpose of feature extraction, and ReLU activation function has been employed due to its inherent low complexity and high computation efficiency; finally, stochastic gradient descent has been used as an optimizer. The main advantage of the current method is that it retains the essential features of the image for prediction along with incorporating a considerable dimensional reduction. The model delivered substantial improvement over existing research in terms of precision, *f*-score, and accuracy of prediction. This model if used precisely can be very effective for healthcare practitioners in determining the thoracic or pneumonic symptoms in the patient at an early stage thus guiding the practitioner to start the treatment immediately leading to fast improvement in the health status of the patient.

## 1. Introduction

The chest carries the vital breath to be dissiminated in to the body parts which provides probably nearly all basic survival elements of the body. A huge number of individuals have been detected annually to suffer from chest ailments of various types on the planet. Tuberculosis (TB), chronic obstructive aspiratory disease (COPD), pneumonia, asthma, and lung disease infections are the most significant chest sicknesses, which have been also considered extremely normal diseases on the planet. Tuberculosis (TB) has been emerging as an omnipresent disease across the globe; this may be evidenced by the fact that in 2017, tuberculosis was responsible for the highest number of unnecessary deaths worldwide [1].

Radiographs popularly known as X-Rays have been used as one of the reliable sources for tracking the vital body parts over the decades. These radiographs have different sequences of evaluation for different body components. For chest X-rays, the evaluation for the lungs, heart, mediastinum, diaphragm, and bony thorax is performed to read the patients' condition while for the abdomen portion, an evaluation of bowel syndrome, psoas and nephritic issues, liver and spleen, and preperitoneal fat lines and a search for unusual calcination are done in order to find the patients' parameters. [2]. The interpretation of chest X-rays is a complex issue due to overlapping of the tissues in the chest area [3].

There is an unprecedented growth in the human progression towards increasing the expectancy of life. Medical Sciences and allied fields of research have made a lot of effort to find resolution for many of the life-threatening diseases. A lot of hard work and research is being done worldwide to make the life of human beings better by finding the best of preventive and diagnostic care. In our current work, we have focused on lung illnesses and proposed the detection through machine learning techniques. As per the Global Burden of Disease Study 2015 [4], approximately 3.2 million people lost lives in 2015 because of chronic obstructive aspiratory illness (COPD), essentially invoked due to smoking and tainting, while 4 million population lost their lives due to asthma. The death data of past is quite alarming and indicative of the toll it may create in coming future generations due to rise in the dominance of various factors which are responsible causes for this disease. Fogel [5] mentions that TB is an irresistible ailment, caused much of the time by microorganisms called Mycobacterium tuberculosis. The microorganisms generally come to the human being by inward breath across the lungs. They outspread from the underlying area within the lungs to different body parts by means of the circulation system, by the lymphatic framework, by means of the aviation routes, or by direct expansion to different organs [6]. COPD is an inflammatory disease of the lung, which causes an obstruction in the flow of air through the lungs; this phenomena is generally progressive and is not reversible [7]. The restriction in air flow through the lungs is normally both dynamic and related with a strange provocative reaction corresponding to the lungs to harmful molecules or vapors. As per clinical reports, the people suffering from COPD encountered breathlessness and cough and abnormal increase in release of mucus, sometimes even accompanied by wheezing. Fergeson et al. [8] stated that asthma is typically a protracted infection described by intermittent assaults of shortness of breath, tightness of the chest, and wheezing. During an asthma assault [9], the coating of the bronchial cylinders swells, making the aviation routes limited and limiting the progression of oxygen within the lungs. The asthma patients generally experience frequent exhaustion, restlessness, decline in the physical activities, etc. As per the Global Burden of Disease Study 2015 [4], asthma has a moderately low casualty rate that contrasted with other interminable sicknesses. The WHO [10] projected that approximately 300 million individuals experience the ill effects of asthma on an average. Asthma is the most widely recognized constant illness among kids. Cancer of the lung (malignancy) is caused due to uninhibited cell development in tissues of the lung [11]. This development may prompt a problem, i.e., spread of the disease from one body part to other body parts like the lungs. By far, most of lung tumors are cancerous for the lung, obtained from endothelium cells or tissues. Lung disease is identified as the most widely recognized cause for disease-related loss of life of human beings and another one generally common in ladies, as per [12]; the disease is liable for loss of 1.76 million humans lives worldwide every year.

With a recent advancement in machine leaning-based processes, it is becoming feasible to detect and diagnose the lung diseases more precisely and well in advance. This may further reduce the causalities originated by these diseases and also the expenditure and consultancy on unessential factors. The true and worthy contribution of the researchers is the dedication of their commendable efforts to help the humans by applying AI to the analyze and forecast chest related disease if any. In the present state of practice, there is a lot of data available freely for research and modelling and also the enhanced computing power available to our machines; it has become very convenient and motivating to develop such systems which help the patients by predicting diseases in advance and help those who are not able to even afford the huge medical bills.

Nowadays, there is an increase in the incorporation of artificial neural network (ANN) structures [13] to develop classification systems for medical diagnosis. The multilayer neural network (MLNN) [14], probabilistic neural networks (PNN) [15], learning vector quantization (LVQ) [16] neural networks, generalized regression neural network (GRNN) [17], and radial basis function (RBF) [18] neural network structures have displayed an evidential improvement over the traditional pattern identification techniques for the diagnose system of the diseases including chest diseases. Various classification systems grounded upon neural network have been employed in chest disease diagnosis stream also. In the past, there have been several neural network-based studies that focused on the chest diseases. The taxonomy of the learning vector quantization neural network structure depends upon the nearness of the unknown information and abovementioned models. A learning vector quantization neural network [16] holds two different layers: one is competitive, and another one is linear output layer. The classification of input vectors is done by the competitive layer. Transformation of the classes of the competitive layer in to the classes of target as described by the user is done by the linear output layer.

The datasets generally used for the classification problems using the techniques like machine learning need the various attributes related to the symptoms, age, sex, snapshot data, X-ray data, and few for specific attributes. By inception of this critical data of the patient, it is easier to train a model and use it for predictive analysis of patients by the health workers in practice. As a practice, medical X-ray images are very often employed for diagnosing few typically subtle human body components including bones, chest, tooth, and skull to name a few. Health experts and workers have eventually relied on this process since the past several decades in order to explore and comprehend fractures and anomalies in human body components. It is pertinent to mention that the X-rays are a very result-oriented diagnostic option in enlightening the pathological variations, further complementing its inherent noninvasive operations and economic viabilities. Abiyev and Ma'aitah [19] demonstrated that the chest-related diseases may be projected in the form of CXR images depicting the cavitation, blunted costophrenic angles, infiltrates, and the consolidations. Upon exploring a typical image of a chest X-ray, it is feasible for a radiologist to evaluate and diagnose certain specific conditions and diseases including effusion, pneumonia, infiltration, bronchitis, cardiomegaly, and fractures [20].

Various researchers have relied on devising methodologies for diagnosis of the chest diseases using the smart and innovative AI-based machine learning methodologies [21]. The detection of prolonged obstructive respiratory and pneumonia infections was devised by inception of the neural systems and an artificial system generating immunity for the environment. For tracking the lung disorders including tuberculosis, pneumonia, and lung disease, chest radiographs are very instrumental. For the purpose of image preprocessing, image segmentation using histogram equalization has been applied. And for the purpose of classification, finally, feed-forward neural networks have been used in the past by the researchers. Though these strategies have been quite helpful in the classification of healthcare-related problems, the deep neural networks outplay these techniques in terms of their efficiency, reliability, and computational time altogether. Many times, to increase the level of accuracy of the classification process, deep neural networks are applied [22]. This is rewarded by deep neural networks with a commendable accuracy outcome. This has led the research community to apply the deep neural networks for classification of medical problems by use of image classification. It has been further evidenced that these networks are able to track and extract classification features which are distinguishing between varies classes of possible states of the evidence of disease. Convolutional neural networks are the favorites when deployed in a deep neural network [23] and have been applied for classification of the medical images; these networks are characterized to possess an ability to different layers of features from the sampled images. Deep convolutional neural networks are recognized for upgrading the diagnostic accuracy and mean squared error for the chest diseases.

In the current research work, convolutional neural networks have been employed on the open dataset from the National Institutes of Health (NIH) which has a huge collection of patient X-ray films for the chest, having a high degree of labelling accuracy. The compilation of the similar work done in the past by other researchers has been given in Section 2, literature review.  Section 3 of the paper gives the complete process of implementing the convolutional neural networks on the dataset used in this study. It gives a stepwise process flow of the whole set of operations performed to generate the model.  Section 4 is the result section, and it shows the finding and achievements of our work and compares them with the related work.  Section 5 provides the conclusion of the work done in this current research and highlights the core outcomes of the current work, the limitations, and future scope of the work.

## 2. Literature Review

Image processing has been an area of interest to the research community for quite a long time, and there are evidences of motivation behind the success that has been achieved in this domain. Thirumaran and Shylaja [24] showcased a brief overview for medical image processing and the various modalities of the process. Khobragade et al. [25] proposed an automated environment catering to the detection and diagnosis of lung diseases explicitly for thoracic diseases with the incorporation of chest radiographs. From the outcomes, it is evidenced that the image preprocessing approaches like equalization through histograms and image processing yield commendable outcomes using the radiograph of the chest. Specified pattern identification, for example, feed-forward artificial neural network, is presenting acceptable outcomes. Chen et al. [26] explored a methodology to boost the dataset considerably. The researcher used an enhanced dataset for training the CNN model for the identification and diagnosis of thorax disease; the model performance was significantly enhanced. They proposed to create a repository of huge collection of images without labelling from clinical services to improvise the performance of their CNN models. Wang et al. [27] attempted to device a “machine-human annotated” wide-range chest X-ray database which reveals the practitioner's medical and technical issues related to the handling of several thousands of the patient databases. They executed a comprehensive quantitative performance standard for a set of eight popular thoracic pathology classification and weakly supervised localization with the deployment of chest X-ray database. The prime objective of research was to device a roadmap for enabling the future efforts to provide aid in promotion of public datasets, which is very critical for this domain of application. Devising a dedicated commercial, robust, reliable, and fully autonomous health diagnosis environment is till date a dream come true. ChestX-ray8 has the potential to equip the data phishing deep neural network models to generate applications which are clinically meaningful which may include instances like pattern mining for some commonly occurring diseases, automation in generating the radiology reports, and analysis correlation of the disease to name a few possibilities. Chan et al. [28] introduced the methodology for segmentation of the lung focused on the abnormal region with the help of numerous overlapping blocks. Texture generated due to computation of multiple overlapping blocks is used to detect the abnormal regions. Concluding this work, the technique efficiently explores lung ailments of the area depicted in chest radiograph image, which further enhances the feasibility of diagnosing the latent issue of the pneumothorax area. Intensity and gradient are the basic fundamentals for texture analysis to detect the pneumothorax. Sharma et al.[29] explored the rib cage area from the lung area using the identification of boundary. To isolate healthy lung area from the cloud of pneumonia Otsu thresholding is incorporated. Despite working on different strategies that may be embraced for thresholding, the pictures of CXR generally yield better outcomes.

After going through the latest research on the feature extraction and use of the same in disease predictions, the current work was motivated. For undertaking the current research work, the objective was to improvise on the existing prediction models and decrease the number of false or erroneous predictions using the machine learning models.  Table 1 summarizes some of the relevant work done by researchers and provided us a strong foundation to generate the initial framework for the experimental process.

## 3. Image Classification Using Convolution Neural Networks

Air pollution has the potential to affect human health both with some direct impact or sometimes indirectly, creating discomfort in physical well-being and resulting in disease or maybe death. Research has evidenced that on exposure of the human body to a polluted environment, there is a sudden rise in the mortality rate [36, 37].

### 3.1. Patient Chest Dataset

Recently, a huge dataset with more than 112120 images of 30805 patients for X-ray lung data was released by the National Institutes of Health [27], for the creation of labels; NLP has been used to convert radiology reports for the classification of the diseases. The approximate accuracy of labelling is more than 90%. The dataset is available for use on data repositories including Kaggle [38]. This dataset inspired the current experimental work on machine learning. In the current work, the authors have undergone an analysis of this chest dataset and then applied machine learning and deep learning for the prediction of a patient to be suffering for any lung ailment; the type of lung ailment and the degree of accuracy of prediction are determined. There are 11 attributes corresponding to the patient in the dataset which include the image index, patient id, patient age, gender, follow-up, label of disease class, view position, image width, image height, pixel spacing-*x*, and pixel spacing-*y*. This project generates a binary classification of the incoming data stream which is basically the patient's individual data pertaining to attributes including patient age, gender, X-ray images, and view position (only the needed attributes have been chosen for modelling), and output is a function that conveys that the patient is suffering from any particular disease or not. This is a relatively new dataset and not much of researchers have explored and presented their work on it.

### 3.2. Convolutional Neural Networks

Convolutional neural networks (CNN) [39, 40] are typically analogous to the artificial neural networks (ANN); they comprise of components called neurons which are capable to optimize on their own through a phenomenon that is called as self-learning. Each neuron of the CNN is capable of receiving at its input some typical input and executes an operation (ranging from a scalar product succeeded by a linear function). The input to this network is a set of raw image vectors, and they are processed to a final output format which is the class score for a particular input vector. Perceptive score weight function is present in this entire network structure spanning all its stages and nodes. Loss functions pertaining to different classes are associated with the terminal layer of the network. Also, all the basic functionalities and modalities of the normal artificial neural networks (ANN) still hold for the CNNs. These networks are specialized for image pattern recognition, and this differentiates them from the ANNs [41]. The classical ANNs suffer from a drawback of low computational efficiency for image-related data due to the complexity in calculations. Additionally, the preprocessing required in a CNN is considerably lesser than other comparable algorithms. A typical convolutional neural network is presented in Figure 1.

The CNN [42] consists of 5 major quantifiable stages. The first stage is the input layer, where the input to the network is supplied in the form of an image. The convolution layer, on its part, convolves the image; i.e., it extracts the significant and differentiating features including edges, colours, and corners from the image received from the previous stage. This layer is multiplied into two matrices, wherein one of the matrices is a known learnable parameter matrix and the other one is the portion of image. The dot product generates a reduced matrix in the end with reduced and required features represented by the matrix, also called as the feature matrix. The pooling layer reduces the feature matrix further in order to generate only dominant image features from the feature matrix. This is done in order to ensure optimized computing efficiency of the system. Average pooling and max pooling are two techniques through which the pooling layer performs this reduction. Till this layer, we reduce the dimensionality of our image. In the fully connected layer [43], the reduced feature matrix is converted to a single vector. The flattened output is sent to a feed-forward neural network [44]; further, back propagation is used during every cycle of training iterations. With maturity of training process, the model is enabled to distinguish certain low-level features and critical features which dominate in images. This felicitates the process of final classification in the output layer. CNNs have been a critical resource in computer vision [29] and image understanding. Generally, the CNNs are realized through a composition of simple linear and nonlinear filters including convolution and rectification, though it becomes a very tedious task to complete them in practice, because the CNNs learn from huge learning datasets, generally, millions of training images, employing intelligent and efficient implementations. Chester explores simple blocks of a CNN in practice, such as convolution, normalisation [45], and pooling [46] which may further be cascaded and drawn out easily to generate CNN architectures. Many of such blocks use optimized CPU and GPU implementations along with CUDA.

### 3.3. Using CNNs in Image Classification

We have taken a stepwise approach to build our model. For the block diagram of Chester, the proposed model for chest disease prediction has been given in Figure 2, initially, the dataset of National Institutes of Health (NIH).

#### 3.3.1. Playing with Data/Analyzing Data

The dataset was loaded using a standard library. After loading, the data is divided into two sections, the one with disease and others having no disease. The various attributes of the dataset are analyzed for any missing values or deviations from the standard format of representing them. Some graph plots were done to understand the basic structure of data and have some idea of correlation among the attributes of similar class data members. We used Matplotlib and Seaborn libraries for the analysis of dataset. There are 15 classes in the full dataset which comprise of one no finding class and other 14 disease classes; since this is a drastically reduced version of the full dataset, some of the classes are sparse labelled as “no findings.” The other 14 disease classes are hernia, pneumonia, fibrosis, edema, emphysema, cardiomegaly, pleural thickening, consolidation, pneumothorax, mass, nodule, atelectasis, effusion, infiltration, and no finding. The images belong to any of these identified classes of disease group.

#### 3.3.2. Preprocessing

In the current work, we have used 40000 image samples out of the total dataset, due to limitation of the hardware to process the huge dataset. After the analysis of data, the data is split up into two sets, one for the purpose of training and the other for testing. We have employed 30000 samples for the purpose of training and 10000 samples for the purpose of testing the model.

#### 3.3.3. Chester

As the next process of the Chester Model, we next transfer the model training dataset and transfer it to further layers of the model. The model comprises of three significant layers in the following order.

*(1) Spatial Transformer Layers*. It further comprises three inherent layers. In the first layer, initially, default routing is transferred, which indicates that the *λ* features of the lung X-ray image correspond to a normal quantum of 0. The next layer is referred to as the batch normalization layer that is responsible for reduction of the amount by which the hidden unit values shift around. Finally, the last layer is the spatial transformer, which corresponds to the removal of maximum significant features for disease classification.

*(2) Extraction of Feature Layers*. For this purpose, the VGG19 model has been pretrained. By default, it loads weight pretrained on ImageNet. There is a group of 19 deep layers where VGG is the feature extraction layer; there are various pretrained classifiers available.

*(3) Classification Layers*. In this case, the first layer defined earlier is used for the purpose of harvesting the VGG19 layers with additional 5 features such as “gender female,” “gender male,” “age,” “view position PA,” and “view position AP.” The purpose of these additional 5 features is to address the issue of sorting. Activation function employed for the current work is Rectified Linear Units (ReLU) [47]. The ReLU activation function was chosen due to its inherent feature of being simpler computationally. The inherent simplicity of ReLU makes it a favorite; here, forward and backward passes are implemented as simple if statements. There is a considerable reduction in cost for training the network using ReLU. This gives the researcher liberty to train larger networks having substantial parameters though maintaining the same computational cost, thereby providing a better capacity to hold and generally greater test set accuracy as well. The mathematical expression given below in equation (1) describes the ReLU function *f* (*x*) for various input values [48].

(1) $$\begin{array}{c} f\left(x\right)=\max\;\left(0,x_{i}\right), \end{array}$$

(2) $$\begin{array}{c} f\left(x\right)=\begin{array}{c} x_{i},\;\text{for }x_{i}\geq 0,\\ 0,\;\text{for }x_{i}<0. \end{array} \end{array}$$

The above equation shows that the ReLU function works well for positive input values and clips the negative values to zero. After creating the model, we define precision, recall, and *f*-score for our case. To optimize the model, we use stochastic gradient descent as an optimizer and pass binary accuracy, precision, recall, and *f*-score as its metrics at different threshold values. Execute the model, and further analyse the model performance. For the purpose of evaluation, stochastic gradient descent (SGD) [49] has been used here, which is a very powerful optimizer. And finally, we ran the model in batches of training (32) and validation (256). The model was run till the 5th epoch. Results were visualized, i.e., testing on images and finding out the possible disease and localizing them, and the model delivered considerable performance.

## 4. Result

The task of analysis of such a huge dataset with X-ray images was very interesting and challenging for us. We could model the system for 40000 images including men and women, selected at random. In the scanned sample of images and from the inferences drawn by our model, it has been analyzed that men are more prone to chest diseases than females. There may be different clinical and behavioral reasons for the same but that is not the scope of our current work. There are various metrics employed for the evaluation of the machine learning models by the researchers. In the current work, we have used the performance evaluation metrics to be precision, recall and *F*-measure for our Chester classifier. The proposed classifier model faired reasonably well and has been well acquainted to this evaluation. Precision refers to the total quantity of positive class predictions which fit to the positive class actually also. Recall refers to the total number of positive class predictions from the complete set of positive instances from the data bank. *F*-measure in turn furnishes with a single score that balances both the issues related to precision and recall represented by a number [50, 51]. Equations (3), (4), and (5) below represent the method to calculate precision, recall, and *f*-score, respectively.

(3) $$\begin{array}{c} \text{Precision}=\text{true}\frac{\text{positive}}{\text{true positive}+\text{false positive}}, \end{array}$$

(4) $$\begin{array}{c} \text{Recall}=\text{TPR}=\text{true}\frac{\text{positives}}{\text{true positives}+\text{false negatives}}, \end{array}$$

(5) $$\begin{array}{c} \text{F}‐\text{score}=\left(1+\beta^{2}\right)\text{precision}*\frac{\text{recall}}{\beta^{2}*\text{precision}}+\text{recall}. \end{array}$$

The current work considered the above metrics for the model evaluation over AUC_ROC and other available metrics due to some of the inherent properties of these metrics that make them more reliable evaluation metrics. The first reason being the fact that the real world data has a tendency to possesses an imbalance among the positive and negative samples. This imbalance has a significant impact on the value of precision but the AUC/ROC do not portray this impact. The ROC/AUC curve has a limitation of not being able to display the performance of the classifier, while in contrast with our used metrics, we can do it with ease.

We have referred to the work of researchers who have previously made their contributions on a similar disease identification with similar dataset or some other datasets. It was a very good foundation for us to get valuable inputs from these already done experimental works.  Table 2 below shows a comparative analysis for work explored by us on the similar data and disease identification problem with same evaluation metrics. Accuracy of our proposed model averages around 80 which is much better than the previous research work being done by the researchers in the same area thus leading to the development of more successful model.

### 4.1. Testing on Images for the Output

For displaying the result of the patient, we used Matplotlib and NumPy library so that we can calculate the result of the X-ray uploaded by the patient or physician. For this, we are segregating the result in separate classes that are in the chest; for the prediction part of X-ray, we have taken a maximum of 4 classes that have the highest values in the X-ray after prediction. As displayed in the images given below in Figures 3 and 4, it can be seen that the result given in NIH dataset as compared with the result produced by our model are accurate and we can tell what the predicted value of diseases beside them is. In the figures below, 4 random cases have been shown for instance. Here, the user, a physician or a patient, filled in the information about X-ray like age, gender, and view position (PA and AP). Basically judging that the patient is ill, before proceeding with the analysis on more important trials, we have chosen prediction score greater than 0.5 to be taken as a threshold. In the given images below, there are various prediction percentages associated with various potential classes of diseases of a patient may have. But as our chosen prediction score is a threshold more than 50, so it will be needed to consider the patient vulnerable for the class of disease where the percentage is more than 50. In Figures 3 and 4, we have analyzed that our model is capable of identifying and classifying even those X-rays that have multiple chest diseases to what percentile it is confident in what disease that the patient might be suffering from and help them in identification of their diseases. These figures lead to the accuracy of the model by detecting the disease which the other models are not able to diagnose.

## 5. Conclusion

Chester is a novel system for analysis and prediction of chest diseases using the profound convolutional systems that is primarily coordinated and permits simple experimentation with clever thoughts. The current work presents a comprehensive mechanism to help the radiologists in diagnosing chest X-rays. This work (Chester) can be utilized as an aide and as an educational tool for students. The framework is intended to process everything locally which guarantees appreciable security. We trust this prompts radiologist to give us criticism which would assist us with improving this instrument and adjust it to their needs. Artificial neural network structures have not been much explored in evaluation of the health issues related to the chest. These examinations have applied distinctive neural system structures to the different chest sicknesses analysis issues utilizing their different datasets. On account of the diverse dataset utilized by the investigations, the immediate correlation of the outcomes was complex. Further, the complexity of the proposed solution is that the current work was very challenging and exciting for the entire team. It is a very complex situation to handle a large volume data, with lakhs of X-ray pictures to scan. The motivation to explore more in the chest disease prediction using the convolutional neural networks for the better disease diagnosis kept the project moving towards its goal. The dataset is not very old, and data is not standardized which makes it difficult to read and map the pictures.

The major outcomes of the research work taken in this paper can be concluded with the following:

1. It has been observed that we can use the neural network structures with some confidence bounds to explore the diagnosis of various chest-related ailments
2. Reasonable results were obtained for the classification of chest diseases using the CNN model
3. The neural networks can self-learn from experience and can be a vital source of help for the practitioners in their diagnostic and treatment efforts

Although we have put our sincere efforts in shaping the current proposed model, with the progression of the work, it was experienced that some more open areas may be addressed to take this work to the next landmark. The modelling may be done with more numbers of epochs, and with parameter tuning, convergence may be achieved conveniently. More degrees of training shall increase the chances of tracking better features to make easier classification. For CNN using VGG, we can experiment on many other pretrained models along with different tweaks that can be made in the model. For the spatial transformer layer, we can try and implement a more complex and sophisticated localization network. The results of the current have fared well to our initial expectations, but to be able to apply it in hospitals, more improvements are needed to increase the precision of the model and also more training data may be employed. Such CNN-based projects tend to employ systems with good computational resources to be able to provide responsive predictions in the minimum possible time to be implementable in practice.

## Figures and Tables

**Figure 1:** A convolutional neural network.

**Figure 2:** Block diagram of Chester—the chest disease predictor.

**Figure 3:** Testing on images for the output.

**Figure 4:** Testing on images for the output.

**Table 1:** Brief summary of inspiration from the earlier research in the domain of disease identification.

S. No.	Author and year	Paper title	Technique used	Objective
1	Bharati & Podder; [30]	Disease Detection from Lung X-ray Images Based on Hybrid Deep Learning Subrato	CNN, vanilla NN	The model proposed classification of chest diseases with its metrics as precision, recall, and *f*-score
2	Rajaraman et al. [31]	Assessment of an Ensemble of Machine Learning Models towards Abnormality Detection in Chest Radiographs	Sequential CNN	Used weighted averaging to in base learners to classify the chest - rays
3	Chan et al. [28]	Effective Pneumothorax Detection for Chest X-Ray Images Using Local Binary Pattern and Support Vector Machine	Support vector machine and local binary pattern	The paper proposed a methodology to detect the lung diseases using the local binary patterns and then further used the SVM technique to classify the type of disease
4	Li et al. [32]	Thoracic Disease Identification and Localization with Limited Supervision	CNN	Identification and localization of abnormalities in the X-rays
5	Sharma et al. [33]	An Analysis Of Convolutional Neural Networks For Image Classification	CNN	The paper focusses on the analysis of real time images of three types of CNN's; these are AlexNets, GoogLeNet, and ResNet50
6	Yao et al. [34]	Learning to diagnose from scratch by exploiting dependencies among labels	LSTM	Used long short-term memory networks for distinction between chest diseases
7	Esteva et al. [35]	Dermatologist-Level Classification of Skin Cancer with Deep Neural Networks	t-SNE-based NN	Analyzed the internal features of the cells by using the CNN with the t-distributed stochastic neighbor embedding
8	Wang et al. [27]	ChestX-ray8: Hospital-Scale Chest X-Ray Database and Benchmarks on Weakly-Supervised Classification and Localization of Common Thorax Diseases	CNN	The work focusses on how thoracic ailments can be discovered and explicitly located with the help of a combined softly supervised multilabelled image sorting and ailment localization framework; the same is verified with the dataset used in the paper

**Table 2:** Comparing our proposed work with existing work on considered metrics.

S. No.	Previous work/model	Precision	Recall	*f*-score	Accuracy
1.	Disease Detection from Lung X-Ray Images Based on Hybrid Deep Learning [30]	0.63	0.69	0.68	0.71
2.	The proposed model for disease prediction	0.77571	0.63098	0.76043	0.80056

## Data Availability

The data used to support the findings of this study are available from the author upon request (gdhiman0001@gmail.com).
